The article "Optimum Feature Selection with Particle Swarm Optimization to Face Recognition System Using Gabor Wavelet Transform and Deep Learning" was retracted in 2024. Reasons: signs of a paper mill; suspected computer-generated content; unreliable results or conclusions; concerns about the data.

# Optimum Feature Selection with Particle Swarm Optimization to Face Recognition System Using Gabor Wavelet Transform and Deep Learning

**DOI:** 10.1155/2021/6621540

**Published:** 2021-03-10

**Authors:** Sulayman Ahmed, Mondher Frikha, Taha Darwassh Hanawy Hussein, Javad Rahebi

**Affiliations:** ^1^ENETCOM, Universite de Sfax, Tunisia; ^2^Kirkuk University, Kirkuk, Iraq; ^3^Department of Software Engineering, Istanbul Ayvansaray University, Istanbul, Turkey

## Abstract

In this study, Gabor wavelet transform on the strength of deep learning which is a new approach for the symmetry face database is presented. A proposed face recognition system was developed to be used for different purposes. We used Gabor wavelet transform for feature extraction of symmetry face training data, and then, we used the deep learning method for recognition. We implemented and evaluated the proposed method on ORL and YALE databases with MATLAB 2020a. Moreover, the same experiments were conducted applying particle swarm optimization (PSO) for the feature selection approach. The implementation of Gabor wavelet feature extraction with a high number of training image samples has proved to be more effective than other methods in our study. The recognition rate when implementing the PSO methods on the ORL database is 85.42% while it is 92% with the three methods on the YALE database. However, the use of the PSO algorithm has increased the accuracy rate to 96.22% for the ORL database and 94.66% for the YALE database.

## 1. Introduction

Face recognition has attracted a lot of interest in recent years [1]. It has become one of the main areas of study in machine vision, pattern recognition, and machine learning. In face recognition, the system selects a face that is more like the desired face according to the trained faces and considers it as the final answer.

Facial recognition was proposed in the 1960s. The first semiautomatic facial recognition system was produced by Woody Bledsoe, Helen Chan Kurt, and Charles Bisson [2]. However, the human face includes a number of details that have been used in many systems, such as artificial age classification [3, 4], facial identification [5], forecasting images and restoration apps [6, 7], description of gender and gestures [8], human-computer interaction (HCI), electronic consumer experience management and audience recording, and tracking of security cameras. Applications for face recognition include monitoring, forensic and medical apps, security applications, in the banks, detection of the person in international centers of transition, access control, and several different fields. Recently, facial recognition technologies were widely used in particular in areas needing strict security measures (airports, police stations, banks, sports fields, and surveillance of entry and exit from business companies).

Computer security is considered to be important in the world today [9]. Face recognition remains an important subject in computer vision sciences. This is because the current systems perform well in relatively controlled conditions but appear to fail when there are issues with facial images, for example, presenting a particular face that differs by various factors, such as variations in posture, position, occlusion, lighting, make-up, and noise- and blur-induced image damage. Although researchers have developed many technologies, multiple different solutions have been attempted to address the problem of changing conditions of the environment. These conditions are the main challenges to facial recognition. Difficulties of the face recognition problem derive from the fact that the faces tend to be approximately similar in their most typical shape (i.e., the front view), and the variations between them are very slight. As a consequence, frontal images formalize a large concentration of the size of the image. This size makes it nearly difficult for typical pattern recognition methods to recognize correctly with a high degree of level of success [10]. Another concentration is the database images [11]. It must have sufficient information for effective face recognition, so the recognition must be possible when dealing with the test image. It is also difficult to determine if there is enough information in the stored images so that the relevant information can be extracted from the databases. Often, unnecessary information is also present in the images of the database, resulting in higher storage consumption and higher processing times. In addition, the optimal size of the images requires to be stored in the databases for effective results [12, 13]. The image size can be compressed to the required size and be stored in the databases. When the image size is compressed, there would be a loss of features, but large numbers of these images can be stored and transmitted through the network fast [14].

In this paper, we used Gabor wavelet transform for feature extraction and then for reducing the features. To find the best feature, the PSO method is used. For the recognition of a face, the deep learning method with 6 layers is used.

## 2. Literature Review

Facial recognition is currently divided into two general categories: appearance-based methods, which statistically process the face, and model-based methods that operate geometrically [15]. For face recognition [16], discriminative dictionary learning and sparse representation are used. In their method, the Gabor amplitude images are implemented by the bank of Gabor filter. Furthemore, the local binary pattern (LBP) is used for feature extraction [17]. Face recognition can be considered one of the most significant applications in the image processing domain [18]. However, illumination and pose invariant recognitions are still the most obvious problems. Viewpoint and illumination are vital to the efficiency of the recognition system because these two factors differ when face images are taken in an uncontrolled environment. Elastic bunch graph matching [19], one of the feature-based methods, has been known for a long time to be accomplished toward several factors such as illumination and viewpoint [18]. Their excessive susceptibility to feature extraction and measurement of the extracted features [20] are what make them unreliable. As a result, the dominant method in the literature is appearance-based methods.

Ahonen et al. proposed a face recognition model with native binary patterns (LBP) [5]. In their study, the point ensuring the robustness of their work is that the algorithm is not sensitive to light.

The fisherface [21] technique is one of the milestones for face recognition under variations. In linear discriminant analysis (LDA), interperson alteration is used optimally with large and intraperson alteration efficaciously small to construct a subspace [21]. Like the PCA [22], the main disadvantage of this technique is that the data space is a consideration of Euclidean. The method does not succeed as multimodal distributed face images when data points are located in a nonlinear subspace.

The sparse representation algorithm based on the Gabor feature is proposed by Yang and Zhang [23]. In their method, the SRC and Gabor features are combined. Using this technique, they improved the human face recognition rate and reduced the complexity of computation.

The deep learning approaches are investigated [24]. The cross-resolution face recognition scenario based on the deep learning method is performed [25]. They robustly extracted the features by deep properties with a cross-resolution scenario. In [26], the angularly discriminative features based on deep learning for face recognition are utilized.

Xu et al. presented the new artificial neural network to face recognition called coupled autoencoder networks (CAN). This helps to overcome age-invariant face recognitions and redemption troubles [27].

The effect of variations in condition on face recognition has been investigated by authors [28]. Consequently, the dominant method has been the appearance-based method. Nikan and Ahmadi [29] introduced a new procedure that propped up fusion of global and local structures.

In [30], local linear transformations were used on behalf of one global transformation, which is a good improvement. The technique suggests different pose classes to different mapping functions. When a probe image is examined, its pose is determined by soft clustering. Deciding the number of pose clusters is a difficult task as in all clustering algorithms. Moreover, novel poses cannot be treated in case of critical variations. In [31], the authors used the neighborhood structure of the input space to determine the underlying nonlinear manifold of multimodal face images. What is used to calculate the basic set is called Laplacian Faces Locality Preserving Projections (LPP). When examining face images with other poses, facial expressions, and illumination conditions, their recognition performance was higher than that of fisherfaces or eigenfaces. In [32], pose variation using view-based eigenfaces was studied. For every view, eigenfaces were numbered to apply a standard dimensional subspace as separate transformations. In addition, a feature-based scheme is included within the eigenfeatures introduced by the authors. As in [33], their performance depends highly on decoupling. Here, the eigenilluminant field technique was used to identify the subspace of poses. Zhao et al. [34] prepared the blurry invariant binary identifier to face recognition. They enhanced the corral among the binary codes of sharp face images and blurred face images of positive image pairs about to learn matrix of projection. Then, they used the learned projection matrix to procure blur-robust binary codes by quantizing projected pixel difference vectors (PDVs) in the trial phase. The discriminative DL method by training a classifier of the coding coefficients is proposed by Mairal et al. [35]. For texture classification and digit recognition, they verified their method. In [36], the sex and country population density interact to predict face recognition talent. The face plus word recognition based on the euro magnetic correlates of hemispheric specialization is presented in [37].

A method that is insensitive to illumination changes was produced by the authors in [38] through combining the generalized concept of photometric stereo and eigenlight field. 3D morphable face models were used in [20, 39, 40, 41] to defined novel poses, which have performances higher than that of the previous research works. Rendering ability for new poses and illumination conditions is exceptional with 3D morphable models [41]. However, the computational cost of generating 3D models from 2D images or using laser scanners to access 3D models decreases the efficiency of the recognition system.

Royer et al. [42] used the eye region to identify a face accurately. The mixed neighborhood topology with the cross decoded patterns is done by [43].

Illumination variance was studied in [44]. The quotient image was suggested by the authors as an identity signature that is insensitive to illumination. While the approximation does not work well, then the probe image has an unexpected shade. Its probe images could be identified with particular illumination then the gallery images. The technique requires only one gallery image for a thing. The technique in [45] introduced additional constraints on the albedo and the surface normal to solve the shadow problem. An illumination cone model was proposed in [20]. The authors discussed a series of images of an object in a fixed pose only describing a convex cone in all lighting conditions. The method needs some images to test their identity and then to guess its surface geometry and albedo map. They defined different illumination cones for each sampled viewpoint to deal with pose variations. The authors discussed in [46, 47] the use of all Lambert reflecting functions to create all kinds of illumination conditions for Lambertian objects. The researchers presented the approximation of plenty of variation of illumination achieved using only nine spherical harmonics. The multiple virtual views and alignment errors are presented in [48]. They manipulated the cross-pose face recognition method.

A methodology for recognition was also used in [46]. In [40], a spherical harmonics approach was exploited, and good recognition results were presented. They designed a 3D morphable model to achieve pose invariance, and this needs to generate 3D face models from 2D images.

Original and symmetrical examples of face training were used [49] to perform collaborative representation for face recognition.

A nonlinear subspace approach was introduced using the tensor representation of faces, such as facial expressions, illumination, and poses [50]. The *n* mode tensor Singular Value Decomposition (SVD) could form the basis of an image. In this technique, various images are required under different variations for each training identity. In [51], there was another nonlinear assumption for each identity in the database, and a gallery manifold is stored. When a test identity with several new poses needs to be defined, first, its probe manifold is constructed, then using manifold to manifold distance can help to define its identity.

The main drawback is the requirement of multiple images of the test person. The authors in [52] introduced a considerable idea by bilinear generative models to decompose orthogonal factors. They showed a separable bilinear mapping between the input space and the lower dimensional subspace. After determining all the parameters of mappings, identity and pose information can be separated explicitly. The recognition and synthesizing capabilities of the technique were analyzed, and the results were encouraging. In [53], illumination invariance was examined using a similar framework. In addition, a ridge regression technique was designed to come through the matrix inversion needed in the symmetric bilinear model. A modified asymmetric model in [54] is aimed at overcoming pose variations. One of the most important factors affecting performance is the solvation of the pose space. The authors in [55] incorporated the nonlinearity of the generative models. They recommended a nonlinear scheme combined with the bilinear model and tried to remove the linearity constraint of the classical generative models. Wright et al. [56] presented a robust method for face recognition. They used sparse representation for feature extraction.

## 3. Proposed Method

In this paper, the face recognition system undergoes stages. These three stages are feature extraction using Gabor wavelet transform, selecting the best features with the PSO method, and face recognition with the deep learning method.

### 3.1. Feature Extraction Using Gabor Wavelet Transform

A much useful instrument in image processing, especially in image identification, is the Gabor filter. The Gabor filter over the spatial field, which has two dimensions, is a Gaussian kernel function as explained below by a complex sinusoidal plane wave:

(1) $$\begin{array}{c} G\left(x,y\right)=\frac{f^{2}}{\pi \gamma \eta }\exp\left(-\frac{{x^{\prime }}^{2}+\gamma^{2}{y^{\prime }}^{2}}{2\sigma^{2}}\right)\exp\left(j2\pi fx^{\prime }+\phi \right). \end{array}$$

Here, *f* represents the sinusoid's frequency, *θ* is the orientation of the normal to the parallel Gabor function's stripes, *ϕ* is the phase offset, *σ* is the Gaussian envelope's standard deviation, and *γ* is the spatial aspect ratio that determines the elliptic support for the function of Gabor.

*x*′ and *y*′ can be calculated as the following equations:

(2) $$\begin{array}{c} x^{\prime }=x\cos\theta +y\sin\left(\theta \right),\\ y^{\prime }=-x\sin\theta +y\cos\left(\theta \right). \end{array}$$

Figure 1 shows the influence of changing some parameters for Gabor's function.

Some of the various benefits of Gabor filters are invariance rotation, scaling, translation, and resistance to distortion of images such as illumination change [58, 59]. They are specially proper for fabric representation plus discrimination.

A range of Gabor filters with other frequencies and directions can be used to extract many features such as texture analysis and segmentation from an image [60]. By varying the orientation, we can look for fabric orientation in a specific direction. By varying the standard deviation of the Gaussian envelope, we change the basis' support or the image's size region being analyzed.

When the features are extracted, the best relative set of features are selected using the PSO method for a flexible face recognition system.

### 3.2. Feature Selection with Particle Swarm Optimization

Particle swarm optimization (PSO) or known as the bird swarm algorithm was initially created in 1995 by Kenny and Eberhart [61]. PSO is a mathematical method that tries to solve optimization problems. For each problem, there are particles (solutions) flying over the problem area based on some mathematical calculations for the velocity and position of the particle. Each particle has fitness values that are measured by the fitness function to be optimized and has velocity that guides the flying of the particles [62].

In computational techniques, PSO is used as a random optimization algorithm for feature selection and classification. This is done by iteratively selecting the most relative and useful set of features to improve or maintain the classification performance for a robust facial recognition system [63].

The basic idea behind this algorithm is the coevolvement of different classes of birds rather than focusing on a certain class of birds. This algorithm contributes to effective search abilities [64]. The PSO algorithm is illustrated in Figure 2.

First, all the particles are assigned primary values; after that, fit values for each particles are estimated. Then, the current fit value is determined; if it is better than the previous one, then we upgrade it to the current value, but if the old fit value is better; we keep it [65]. The algorithm ends, and this process is repeated until the best solution is obtained.

The equation of the PSO algorithm is demonstrated below:

(3) $$\begin{array}{c} v_{i}^{d}\left(t+1\right)=wv_{i}^{d}\left(t\right)+c_{1}r_{1}\left(p{\text{best}}_{i}^{d}\left(t\right)-x_{i}^{d}\left(t\right)\right)+c_{2}r_{2}\left(g{\text{best}}^{d}\left(t\right)-x_{i}^{d}\left(t\right)\right). \end{array}$$

Each particle is upgraded with two “best” values in each iteration. Here, *v* denotes velocity which is bounded between *w*_max_ and *w*_min_, *w* is inertia weight, and *x* is solution [66, 67]. Continuing, *t* refers to the number of irritation, *i* to the order of practicality in population, and *d* to the dimension of search space. *c*_1_ and *c*_2_ indicate acceleration factor; *r*_1_ and *r*_2_ are two independent random numbers in [0, 1]. *p*best implies the personal best solution (the best solution that has been found yet), while *g*best implies the global solution which is recorded by the particle swarm optimizer. This optimizer is the best worth yet achieved by any particle for the entire population.

Afterwards, velocity is updated to a probability value as demonstrated in the following equation:

(4) $$\begin{array}{c} s\left(v_{i}^{d}\left(t+1\right)\right)=\frac{1}{1+e^{\left(-v_{i}^{d}\left(t+1\right)\right)}}. \end{array}$$

Practical position and *p*best with *g*best are converted to the following equations:

(5) $$\begin{array}{c} x_{i}^{d}\left(t+1\right)=\left\{\begin{array}{cc} 1, & \text{if }\mathrm{rand}<s\;\left(v_{i}^{d}\left(t+1\right)\right),\\ 0, & \text{otherwise}, \end{array}\right. \end{array}$$

where rand is a random number between 0 and 1.

(6) $$\begin{array}{c} {p\text{best}}_{i}\left(t+1\right)=\left\{\begin{array}{cc} x_{i}\left(t+1\right), & \text{if }F\left(x_{i}\left(t+1\right)\right)<F\;\left({p\text{best}}_{i}\left(t\right)\right),\\ {p\text{best}}_{i}\left(t\right), & \text{otherwise}, \end{array}\right.\\ {g\text{best}}_{i}\left(t+1\right)=\left\{\begin{array}{cc} {p\text{best}}_{i}\left(t+1\right), & \text{if }F\left({p\text{best}}_{i}\left(t+1\right)\right)<F\;\left({g\text{best}}_{i}\left(t\right)\right),\\ {g\text{best}}_{i}\left(t\right), & \text{otherwise}, \end{array}\right. \end{array}$$

where *F* is the fitness function:

(7) $$\begin{array}{c} w=w_{\max}-\left(w_{\max}-w_{\min}\right)\left(\frac{t}{T_{\max}}\right). \end{array}$$

The parameter used for particle swarm optimization is shown in Table 1.

We obtained these parameters experimentally.

### 3.3. Convolutional Neural Network

The main component of a convolution neural network (CNN) is the convolution layer. The approach behind a convolution layer is a feature which has been learned locally for any given input (for example, any 2D images). It should be helpful in other regions of that same input source. For example, a feature for edge detection, which was proved useful in one part of the image, might be helpful in the other regions of the image at a possible general feature extraction stage. The learning of other features in an image such as edges oriented at an angle or curves is obtained by sliding the filters across the image with a step or stride size which is constant for a given convolution layer.

Layers of more than one subsampling and convolutional layer, preferably fully added layers, are called CNN. *M* is the height and width of the image, and *r* is the number of channels, while the input of an accessible layer is the image *m* × *m* × *r*, e.g., an RGB image has *r* = 3. The convolutional layer can differ in every core it has; this is because it will have *k* kernels or filters of size *n* × *n* × *q*, where *n* is much smaller than the size of the image and *q* could be smaller than the number of channels.  Figure 3 shows the general topology of a CNN.

## 4. Experimental Result and Discussion

This chapter shows that the outcomes are derived from the simulation using MATLAB 2020a. The recognition system consists of three stages. The first is *the feature extraction*; in this stage, we used Gabor wavelet transform. The second is *feature selection*. In this stage, we used particle swarm optimization (PSO), on features that are obtained from Gabor wavelet transform. In the final stage, *the classification*, we used deep learning with 6 layers.

The database in this study is used from ORL databases. The ORL (Olivetti Research Laboratory) face database contains 400 images of 40 different people. There are ten different grayscale images of each of 40 distinct persons. Images were captured at various times, and they have various variations including various expressions (closed/open eyes, not smiling/smiling). The details of the face (with/without glasses) are included. Images were taken with a tolerance for some tilting and rotation of the face up to 20 degrees [49].

Some face images from the ORL database are shown in Figure 4.

Some simulation of the first face image is implemented on MATLAB 2020a, and the results are shown in Figure 5.

For evaluating the proposed method, we used the mean squared error (MSE), mean absolute percentage error (MAPE), and *R*-squared method. The mean squared error (MSE) is shown by

(8) $$\begin{array}{c} \text{MSE}=\frac{1}{n}\overset{n}{\underset{i=1}{\sum }}{\left(Y_{i}-\overset{\wedge }{Y_{i}}\right)}^{2}. \end{array}$$

The mean absolute percentage error (MAPE) is shown in the following equation:

(9) $$\begin{array}{c} \text{MAPE}=\frac{1}{n}\overset{n}{\underset{t=1}{\sum }}\left|\frac{A_{t}-F_{t}}{A_{t}}\right|. \end{array}$$

For *R* square, we have the estimated value as

(10) $$\begin{array}{c} \overset{¯}{y}=\frac{1}{n}\overset{n}{\underset{i=1}{\sum }}y_{i}. \end{array}$$

Then, the variability of the data set can be measured using three sums of squares formulas. The total sum of squares is proportional to the variance of the data:

(11) $$\begin{array}{c} SS_{\text{tot}}=\underset{i}{\sum }{\left(y_{i}-\overset{¯}{y}\right)}^{2}. \end{array}$$

The regression sum of squares is also called the explained sum of squares:

(12) $$\begin{array}{c} SS_{\text{reg}}=\underset{i}{\sum }{\left(f_{i}-\overset{¯}{y}\right)}^{2}. \end{array}$$

The sum of squares of residuals is the residual sum of squares:

(13) $$\begin{array}{c} SS_{\text{res}}=\underset{i}{\sum }{\left(y_{i}-f_{i}\right)}^{2}=\underset{i}{\sum }e_{i}^{2}. \end{array}$$

The most general definition of the coefficient of determination is

(14) $$\begin{array}{c} R^{2}\equiv 1-\frac{SS_{\text{res}}}{SS_{\text{tot}}}. \end{array}$$

Table 2 shows the specifications of the layer that is used in deep learning.

The procedure and test were performed using actual with symmetrical species from ORL and YALE datasets. The results are shown in Figures 6–9. The results show that the system using the ORL dataset revealed how the preprocessing stage improves the accuracy. They also indicate how we can merge or fuse two methods of feature extraction to produce a powerful third method that can accomplish the job.

The comparison of the MSE, RMSE, MAPE, and *R* for train data is shown in Figure 7.

The result using the PSO is shown in Figures 10–13.

We have observed that the recognition rate and accuracy results from the experiments cannot be met when utilizing the Gabor wavelet and deep learning due to some variation of the values of features which corrupts the classification step. So, when compared with Gabor wavelet features, the variety will be large. Hence, the features are between -14 and 254. Therefore, optimum features are chosen.

PSO methods try to address this problem by selecting only the optimum features from Gabor wavelet. The performance of the classifier is based on the number of features. Too less or too redundant features can reduce the accuracy rates. Therefore, the number of features must be chosen carefully. In PSO, the basic process is that there are a number of particles; each one of them is flying through the problem area arbitrarily searching for the previous best solution and the global best solution of the whole swarm. Then, velocity is modified at each iteration which will define the movement of the particles to be more or less random. Therefore, the algorithms are converged. This method was used in literature [68], using the PSO method for selecting the best features.

In our experiments, we have used Gabor wavelet for feature extraction obtaining 10304 features. When the features were extracted, the implementation of PSO reduces the features to 5142. The best and most optimum features are selected by eliminating the highest and lowest values of features using the fitness function which determines the features that are the closest to each other in the amount. The experimental results obtained a 96% recognition rate on the ORL database when implementing the proposed method.

For the cause of completeness, we compare the performance of PCA [22], SRC [56], CRC [69], Gabor wavelet with Euclidian method [57], symmetrical face sample method [49], and the proposed method.

The comparison of other methods with the proposed methods is shown in Table 3.

## 5. Conclusion

The use of the symmetry property of the face is an efficient way to increase the performances of the face recognition systems. In this study, a new method is provided for the face recognition system. The new method is upgraded to use the benefits of symmetry property in the face data. The feature space is another way to implement the use of symmetry property in the face. There are many methods for feature extraction; however, none of them can handle the symmetry procedure in the feature space. The suggested methods can perform the symmetry procedure either in the image space or in the feature space. The introduced method is examined and tested for face recognition using data from ORL and YALE datasets.

## Figures and Tables

**Figure 1:** (a) Different values of wavelength (left: 25, right: 50), (b) different orientation (left: 0, right: 45), (c) changing the values of phase shift (left: 180, right: 90), (d) aspect ratio very large (left) and very small (right), and (e) different bandwidth values (left: large, right: small) [57].

**Figure 2:** Particles searching for the best and optimum solution: (a) first iteration and (b) last iteration.

**Figure 3:** CNN's topology.

**Figure 4:** ORL database.

**Figure 5:** (a) Real image, (b) left side, (c) right side, (d) left side's mirror, (e) right side's mirror, (f) integration of left side with mirrors, and (g) integration of right side with mirrors.

**Figure 6:** Train result.

**Figure 7:** The comparison of the MSE, RMSE, MAPE, and *R* for train data.

**Figure 8:** Test result.

**Figure 9:** The comparison of the MSE, RMSE, MAPE, and *R* for test data.

**Figure 10:** Train result with PSO.

**Figure 11:** The comparison of the MSE, RMSE, and *R* for train data.

**Figure 12:** Test result with PSO.

**Figure 13:** The comparison of the MSE, RMSE, and *R* for train data.

**Table 1:** Parameter for particle swarm optimization to select the best features.

Parameter	Description	Value
*N*	Number of particles (population size)	40
*T*	Maximum number of iterations	15
*c*_1_	Cognitive factor	3
*c*_2_	Social factor	2.5
*w*_max_	Maximum bound on inertia weight	0.8
*w*_min_	Minimum bound on inertia weight	0.5
*V*_max_	Maximum velocity	5

**Table 2:** Specifications of the deep learning.

	Type	Activation	Learnable
1	Sequence input	5141	—
2	LSTM	200	Input weights (800∗5141) Recurrent weights (800∗200) Bias (800∗1)
3	Fully connected	50	Weights 50∗200 Bias 50∗1
4	Dropout	50	—
5	Fully connected	1	Weights 1∗50 Bias 1∗1
6	Regression output	—	—

**Table 3:** Comparing other methods with the proposed methods.

Method	Recognition rate
PCA [22]	53.2%
SRC [56]	75.12%
CRC [69]	79.4%
Gabor wavelet with Euclidian method [57]	83.44%
Symmetrical face sample method [49]	81.43%
Proposed method	85.25%

## Data Availability

All data available for readers are included within the article.
